The article "Insight into the Effects of High-Altitude Hypoxic Exposure on Learning and Memory" was published in 2022. Journal: Oxid Med Cell Longev.

# Insight into the Effects of High-Altitude Hypoxic Exposure on Learning and Memory

**DOI:** 10.1155/2022/4163188

**Published:** 2022-09-14

**Authors:** Zi-ang Zhang, Yafei Sun, Ziyan Yuan, Lei Wang, Qian Dong, Yang Zhou, Gang Zheng, Michael Aschner, Yuankang Zou, Wenjing Luo

**Affiliations:** ^1^School of Aerospace Medicine, Fourth Military Medical University, No. 169 Chang Le West Rd., Xi'an, Shaanxi 710032, China; ^2^Department of Occupational and Environmental Health, The Ministry of Education Key Lab of Hazard Assessment and Control in Special Operational Environment, School of Public Health, Fourth Military Medical University, No. 169 Chang Le West Rd., Xi'an, Shaanxi 710032, China; ^3^Institute of Medical Information and Library, Chinese Academy of Medical Sciences and Peking Union Medical College, Beijing 100020, China; ^4^Department of Biochemistry and Molecular Biology, School of Basic Medicine, Fourth Military Medical University, No. 169 Chang Le West Rd., Xi'an, Shaanxi 710032, China; ^5^Department of Molecular Pharmacology, Albert Einstein College of Medicine, Bronx, NY 10461, USA

## Abstract

The earth land area is heterogeneous in terms of elevation; about 45% of its land area belongs to higher elevation with altitude above 500 meters compared to sea level. In most cases, oxygen concentration decreases as altitude increases. Thus, high-altitude hypoxic stress is commonly faced by residents in areas with an average elevation exceeding 2500 meters and those who have just entered the plateau. High-altitude hypoxia significantly affects advanced neurobehaviors including learning and memory (L&M). Hippocampus, the integration center of L&M, could be the most crucial target affected by high-altitude hypoxia exposure. Based on these points, this review thoroughly discussed the relationship between high-altitude hypoxia and L&M impairment, in terms of hippocampal neuron apoptosis and dysfunction, neuronal oxidative stress disorder, neurotransmitters and related receptors, and nerve cell energy metabolism disorder, which is of great significance to find potential targets for medical intervention. Studies illustrate that the mechanism of L&M damaged by high-altitude hypoxia should be further investigated based on the entire review of issues related to this topic.

## 1. Introduction

Oxygen is essential for human metabolism and physiological function maintenance. However, approximately 400 million people working and living at terrestrial altitudes above 1500 meters are exposed to short- or long-term hypoxia. As the partial pressure of oxygen drops sharply as the altitude increases, maintaining a stable oxygen environment in the body is crucial.

The article "Insight into the Effects of High-Altitude Hypoxic Exposure on Learning and Memory" was published in 2022. Journal: Oxid Med Cell Longev.

Exposure to hypoxia results in many physiological changes. The brain shows to be more sensitive to the fluctuation of oxygen content, which consumes about one-fifth of the entire body's oxygen. Therefore, a hypoxic environment affects brain function, and even a short exposure to hypoxia may cause irreversible damage [1, 2]. The incidence of hypoxic brain injury caused by perinatal asphyxia is 1‰ to 6‰, and 25% to 30% of survivors have long-term sequelae, including various degrees of decline in learning and memory function [3, 4]. It is believed that the longer the exposure to hypoxia, the greater the damage [5, 6]. In addition to impaired cognitive physiology and psychological function, brain damage caused by hypoxia may also lead to learning and memory (L&M) defects. An extended period of hypoxia may be sufficient to change a brain's structure [7]. There are many transcription factors and regulatory proteins involved in the homeostatic regulation of optimal oxygen environment, including hypoxia-indubitable factor (HIF).

Previous research has shown that people living on plateaus with an average elevation of more than 2,000 m above sea level have developed unique adaption over time. For example, the blood flow and brain blood flow velocity are higher for Tibetans living on the Qinghai-Tibet plateau than those on the plains [8, 9]. The purpose of this review is to summarize the pertinent research progress of hypoxia's effects on L&M and provide references for the prevention and treatment of cognitive impairments and related situations caused by hypoxia.

## 2. Plateau Hypoxia Environment

The plateau covers over 45% of the earth's land area. As the highest plateau in the world, the Qinghai-Tibet plateau has an average altitude of more than 4,000 meters, and an atmospheric oxygen partial pressure is lower than 40% compared to that of the sea level. Aside from its low temperature, intense radiation and large temperature differences between day and night make the Qinghai-Tibet plateau a harsh place to live [10]. Expose to high altitude hypoxia environment, our body will undergo series of adaptions: number of red cells and level of hemoglobin concentration and hemoglobin oxygen dissociation (P_50_) will be upregulated, while frequency and depth of breathing and arterial oxygen saturation will be downregulated [11, 12]. If these changes exceed the range of biological adaptation, then damage to many organ systems, including the central nervous system (CNS), will appear. On the Qinghai-Tibet plateau, a large number of indigenous people, namely, the Tibetans, have lived in the low-oxygen environment for generations and thus adapted physiological changes. Compared to those who have inhabited in the plains for decades, the Tibetans have a significant higher concentration of P_50_, and their hemoglobin levels are lower [11, 13]. Furthermore, their blood flows faster intend to maintain oxygen supply [8].

The article "Insight into the Effects of High-Altitude Hypoxic Exposure on Learning and Memory" was published in 2022. Journal: Oxid Med Cell Longev.

### 2.1. Hypoxia and Organ System Impact

Many studies on the Tibetans and their close relatives Sherpa have shown that specific variant in endothelial PAS Domain Protein (EPAS1) is an early adaptation signal to hypoxia [14, 15]. Additionally, the Tibetans have highly differentiated haplotypes of this protein [16, 17]. The EPAS1 gene expression levels may be associated with lower hemoglobin concentrations [12, 18]. Another gene that has attracted widespread attention is Egl nine homolog 1 (EGLN1), which encodes proline hydroxylase 2 (PHD2). The EGLN1 mutations in Tibetans lead to increased degradation of HIF in the body under hypoxia conditions, thereby preventing the production of excessive red blood cells and reducing the risk of prenatal death, heart disease, and stroke [19–21]. Even though the Tibetans have adapted to the plateau environment, they could still suffer from the effects of hypoxia on the plateau. Based on an analysis of a large number of Tibetan residents, researchers found that residents are more likely to develop depression than those living on the plain [22]. Plateau hypoxia also affects drugs metabolism in the body. For example, people living in plateau regions often need to intake higher doses of streptomycin to treat infections [23]. As hypoxia research continues, the impacts of plateau hypoxia environment on multiple organs and systems have gained researchers' wide attention [24–28]. The influence of hypoxia on organ and systems is briefly listed in Table 1.

### 2.2. Hypoxia and Hypoxia-Inducible Factors

The hypoxia-inducible factors, comprised of an O_2_-sensitive *α*-subunit (mainly HIF-1*α* and HIF-2*α*) and a constitutively expressed *β*-subunit, are key transcription factors mediating adaptive responses to hypoxia and playing a vital role in coping with ischemia. Under normal oxygen concentration, HIFs have a short half-life, and the hydroxylation of two specific proline residues in the HIF-*α* chain promotes its interaction with VHL E3 ligase, which in turn causes ubiquitination, leading to HIF-*α* proteasome destruction. However, under hypoxia environment, HIF degradation is inhibited, and gradual accumulation of the factors happens. HIF-*α* enters the nucleus, dimerizes with HIF-*β*, and then binds with hypoxia response elements (HREs). The stability of neuronal cell function requires the effective participation of HIF. The HIF family is involved in regulating the expression of genes related to physiological activities, cell metabolism, and survival [19, 29–31], and those processes lead to cell adaption to the hypoxia environment. HIF promotes the expression of glycolysis-related enzymes by reducing cell division and inhibits the phosphorylation of pyruvate dehydrogenase (PDH) to mediate the conversion of the body's metabolic pathways from oxidative phosphorylation to glycolysis and improve adaption to hypoxia [19, 32, 33]. In addition, HIF-1*α* increases blood vessel density and increases oxygen diffusion distance by activating the expression of angiogenic genes, thereby enhancing the body's tolerance to hypoxia [34]. Recent studies have found that inhibiting the accumulation of HIF-1*α* reduces angiogenesis, activates glia, and aggravates oxidative damage in the hippocampus, and the above changes will later on lead to L&M disorders [35]. HIF-1*α* has been shown to increase the expression of vascular endothelial growth factor (VEGF), a key regulator of physiological angiogenesis, and reduce the damage by inhibiting the expression of cysteine-aspartic protease 3 (caspase-3) and some cytokines such as interleukin-6 (IL-6) [36–38].

The article "Insight into the Effects of High-Altitude Hypoxic Exposure on Learning and Memory" was published in 2022. Journal: Oxid Med Cell Longev.

As the research progresses, the function of HIF-2*α*, a product of the EPAS1 gene, has raised significant concerns. Despite the structural similarity of HIF-2*α* to HIF-1*α* [39], HIF1*α* plays a greater role in regulating metabolic reprogramming, whereas HIF2*α* transcription primarily regulates a diverse subset of transcription factors and coregulators that contribute to its diverse roles in hypoxia. At high oxygen levels, HIF-2*α* is more stable than HIF-1*α*, whereas HIF-1*α* is more active in short (2-24 hrs) and high-intensity anoxic environments (<0.1% O_2_), while HIF-2*α* is more stable in prolonged and mild hypoxia environments [40]. HIF-2*α* is mainly expressed in astrocytes, while HIF-1*α* prefers accumulating in neurons [38, 41]. HIF-2*α* in astrocytes can regulate L&M by affecting synaptic plasticity [42, 43], while HIF-1*α* mediates the transcriptional expression of metabolic genes in astrocytes [41]. We believe that the specific expression pattern of hypoxia-inducible factors in nerve cells may be related to the rate of cell metabolism adapting to the change of O_2_ concentration. VEGF and erythropoietin (EPO) as the target genes of HIF have been discovered to regulate vascular dynamics in organ systems, including the central nervous system. HIF can stimulate the expression of VEGF and increase angiogenesis [44]. EPO is derived from liver parenchymal, and tubulointerstitial cells are involved in the process of perception of the hypoxia environment and hypoxia signal transduction, activating the signal transducer and activator of transcription 3 (STAT3) [45], increasing the expression of antioxidant enzymes, and reducing the production of reactive oxygen species as well [46]. In addition, EPO may promote brain-derived neurotrophic factor (BDNF) synthesis affecting synaptic plasticity in long-term memory [47, 48]. HIF-2*α* exerts a stronger effect on EPO generating than HIF-1*α* does [49]. Studies have shown that only by simultaneously knocking out both HIF-1*α* and HIF-2*α* would there be a significant inhibitory effect on the production and transcription of EPO [50]. In short, HIFs are important for hypoxic stress in neurons and affect downstream signal transduction pathways, whereas the mechanism of target gene divergency of HIF-1*α* and HIF-2*α* remains to be understood (Figure 1).

The article "Insight into the Effects of High-Altitude Hypoxic Exposure on Learning and Memory" was published in 2022. Journal: Oxid Med Cell Longev.

## 3. Hippocampus and L&M

Learning is defined as the acquisition of knowledge through experience or exploration, while memory is defined as the process of retaining newly acquired information over time. Memory can be divided into sensory memory, short-term memory, and long-term memory [51]. Learning and memory (L&M) are interconnected and mutually influenced. The hippocampus, one of the fragile and slender structures located at the bottom of the medial temporal lobe, is an integrated center of L&M. The hippocampus is very vulnerable to ischemia, hypoxia, inflammation, and epilepsy [52, 53]. Anatomically, the hippocampus is composed of different subregions, including cornu ammonis 1 (CA1) and cornu ammonis 2 (CA2). Even limited hippocampal damage can lead to impairment of memory function [53, 54]. Scoville and Milner once reported that Henry Molaison, a patient without hippocampus, had clinical symptoms of recent memory loss but with nondeclarative memory intact. This indicated that this structure is vital for memory storage, but not related to nondeclarative memory [55].

The processing of episodic memory requires the involvement of the entorhinal-hippocampal network. Different subregions of the hippocampus play various types of functions in L&M. The CA1 subregion, which is closely linked to the subicular complex, is closely related to spatial memory [56, 57], and they are jointly responsible for visual and speech memory. Alzheimer's disease (AD) patients with hippocampal atrophy commonly suffer from speech memory disorders [58]. CA2, an important center for social cognitive memory processing, and dentate gyrus (DG) are more closely related to short-term and intermediate memory, while CA1 is closely related to long-term memory [59, 60]. CA3 and DG are important in memory coding and early retrieval [61], and CA1 occupies a more important position in consolidation and late retrieval [62]. The prefrontal cortex interacts with the hippocampus to participate in memory processing and integration processes, which is conducive to the generalization of cross-knowledge domains [63, 64]. In the matter of learning, recent studies have speculated that the anterior part of the hippocampus can dispose of novel decision-making schemes based on previous experience [63]. Nonetheless, the traditional view does not agree on the hippocampus' role in progressive stimulus-response and value-added learning. In the most recent researches, the CA1, CA2, and CA3, but not DG, have shown to be important for value-added learning [65]. The hippocampus is also significant for statistical learning [66]. Hippocampus-dependent L&M is not inherent but parallel to the development of human beings. Certain sensory signals trigger neuronal activities. These activities are important for brain development which is necessary for synaptic connectivity of the network. But how hippocampal-dependent L&M formation during development remains as a difficult neurobiological issue incorporating complex interactions between neuronal networks.

The article "Insight into the Effects of High-Altitude Hypoxic Exposure on Learning and Memory" was published in 2022. Journal: Oxid Med Cell Longev.

Besides, other parts of the brain are also involved in L&M. For example, the striatum is associated with habitual learning and progressive stimulus responses, the amygdala participates in the acquisition of emotional behavior [67, 68], and the temporal cortex is sensitive to hierarchical features of memories [69, 70]. In general, the limbic system is the core brain region adopted in L&M. As a crucial part of the limbic system, different subregions of the hippocampus play different functions in L&M.

## 4. Synaptic Plasticity

A cluster of neurons interact to form neural circuits through synapses, and recent findings have strongly supported that synaptic plasticity is the neurobiological basis of L&M [71, 72]. Synaptic plasticity involves structural plasticity and functional plasticity. Structural plasticity refers to the activity-dependent change of dendritic spines and their internal substructures [73]. Once stimulated, synaptic spines are either highly contracted or extended. Functional plasticity includes long-term potentiation (LTP) and long-term depression (LDP), which store large amounts of information by selectively enhancing or weakening synaptic connectivity [74]. Presynaptic nerve fibers are given high-frequency stimulation, resulting in enhancement of excitatory postsynaptic potential (EPSP) in postsynaptic cells. This phenomenon is reported as LTP, which is generally considered as a sign of neuron storing information. LTP increases the density of synapses and the diameter of dendritic spines in synapses, whereas long-term depression (LTD) leads to the contraction of dendritic spines. Synaptic morphological modifications are the anatomical basis for synaptic functional changes. Environmental stimuli result in dendritic spine structural changes, and the new neural environment formed by this change allows the body to participate in certain behaviors, such as learning [75]. LTP collectively controls the generation and shaping of memory. LTD is a negative modulation of long-term memory, a prolonged-term reduction in synaptic transmission performance. It is manifested by reduced release of glutamate and decreased expression of the N-methyl-D-aspartic acid (NMDA).

The article "Insight into the Effects of High-Altitude Hypoxic Exposure on Learning and Memory" was published in 2022. Journal: Oxid Med Cell Longev.

NMDA receptors are a key link in the induction of LTP and are also considered as an important molecular basis for L&M. Under normal conditions, the glutamate (Glu) released by the presynaptic membrane is unable to bind to the NMDA receptor, which is normally blocked by Mg2^+^. Instead, glutamic acid binds to *α*-amino-3-hydroxy-5-methyl-4-isoxazole propionic acid (AMPA) receptor of the postsynaptic membrane, causing Na^+^ influx and formation of postsynaptic membrane depolarization. The reduction of the blocking effect caused by Mg2^+^ on NMDA receptors is also seen. Then, depolarization causes Ca^2+^ influx and leads to LTP. Postsynaptic membrane depolarization simultaneously induces intracellular Ca^2+^ release, resulting in increased intracellular Ca^2+^ concentration. And Ca^2+^, an intracellular signaling molecule, activates the expression of calcium-CaM-dependent protein kinase II (CaMK II) and increases the phosphorylation level of NMDA receptors, in doing so increases synaptic signal delivery efficiency. Studies have found that excessive activation of NMDA receptors gives rise to a large influx of Ca^2+^ and prompts neuron damage. The entire process leads to a decline in L&M levels [76].

In recent years, the investigation has revealed that the ubiquitin-proteasome pathway (UPP) plays a crucial role in regulating the expression of presynaptic and posterior membrane proteins. The latter proteins take part in nerve impulse transmission and synaptic plasticity. After ubiquitin binds to its substrates, it starts being degraded by protease. The connection between ubiquitin and protein depends on three enzymes E1, E2, and E3, among which, E3 determines the specificity of the substrate [77]. Studies have indicated that in the rat hippocampus, proteasome activity is essential for the formation of LTD [78]. Other evidence has shown that the precise coordination of protein synthesis and proteasome-mediated protein degradation is fundamental for the regulation of mGluR-dependent LTD production [79].

The article "Insight into the Effects of High-Altitude Hypoxic Exposure on Learning and Memory" was published in 2022. Journal: Oxid Med Cell Longev.

## 5. Impaired L&M Caused by Hypoxia Environment at High Altitude

Previous report has indicated that after acute exposure to a 4,200 m high altitude environment for 3 days, the L&M abilities of rats were severely affected [80]. 18 healthy young men were exposed to levels of 2,800 m, 3,600 m, and 4,400 m at low pressure and hypoxia chambers for an hour, respectively. Results indicated that short-term memory decreases with increased altitude [81]. Evidence from pilots and aircrews showed that a high-altitude environment causes altered cognition by interfering with new memory coding but not with memory retrieval [82]. Other studies have also found that exposing zebrafish to hypoxia environments significantly impairs learning [83]. However, Wittner and Riha found that short-term acute hypoxic exposure could improve spatial memory ability, and intermittent hypoxia can significantly enhance the spatial L&M ability of mice [84]. This phenomenon may be relevant to the escalation of the small regulatory polypeptide of amino acid response (SPAR) expression in the hippocampus [85]. Previous studies have shown that acute and chronic hypoxia can lead to increased oxidative stress response level of cerebral cortical cells, enhance cell autophagy, trigger neuronal excitability toxicity reaction, and aggravate apoptosis and brain function damage [86, 87]; the process may be related to the lysosome membrane permeability change [87], but this review focuses on hypoxia damage in the hippocampus.

### 5.1. Hypoxia and Apoptosis of Hippocampal Neurons

Different subregions of the brain tolerate different degrees of hypoxia, where the “anoxia-prone cells” are brainstem neurons and hippocampal CA1 vertebral neurons [88]. There is evidence showed that hypoxia stimulates the expression of cellular oncogene fos (c-fos) in the hippocampus, and c-fos protein can be treated as a marker of neuronal activation by nociceptive stimuli [88]. Under hypoxia conditions, a reduced expression of GAD protease in hippocampal neurons leads to changes in inhibitory synaptic density [89]. Moreover, others have found that the density of dendritic spines in neurons of CA1 area decreases after hypoxic exposure [90], and the apoptosis in this area increased significantly. Additional research has illustrated that the activity of caspase-3 in CA1 neurons increased [86] and hypoxia-activated p53 protein expression through multiple pathways, leading to neuronal apoptosis [91]. Analysis of the transcriptome data has revealed that the imbalance of miR-26b and miR-207 expression played a role in the process of cognitive impairment caused by hypoxia [92]. In addition to the CA1 subregion, the effects of hypoxia on CA3 cannot be ignored. In hypoxic environments, lipofuscin particles deposit in CA3 area, resulting in a gradual accumulation of damaged macromolecules and further inducing morphological changes of hippocampal mitochondria in memory-impaired mice. Nonetheless, Tsai et al. have shown that intermittent hypoxia intervention after cerebral ischemia can trigger hippocampal neurogenesis and synaptic reformation, which may be related to the activation process of BDNF expression [93]. Furthermore, hydrogen can also activate protein kinase B (AKT) by reducing the expression of miR-200a-3p, miR-200b-3p, or mir-429, thereby reducing apoptosis in hippocampal neurons [94].

The article "Insight into the Effects of High-Altitude Hypoxic Exposure on Learning and Memory" was published in 2022. Journal: Oxid Med Cell Longev.

### 5.2. Hypoxia and Dysfunction of Hippocampal Neurons

It has long been understood that hypoxia impairs brain function in both humans and animals. Human short-term memory performance will be deteriorated after short-term exposure to acute, mild, and moderate hypoxia, and these effects become much worsen with higher altitude. Therefore, neuronal dysfunction caused by acute hypoxia deserves widespread attention compared to neuronal death caused by chronic severe hypoxia.

#### 5.2.1. Hypoxia and Oxidative Stress in Neurons

Hypoxia-induced oxidative stress in neurons can lead to structural changes in protein and inflammation and ultimately affect nervous system function [95–97]. Microglia, which can differentiate into proinflammatory (M1) and anti-inflammatory (M2) cells [98, 99], are involved in immune effects after nervous system injury. Under physiological conditions, microglia are functionally involved in immune defense and cell debris cleanup. When stimulated by neurotoxic substances, such as interleukin (IL) and interferon (INF), microglia activate and transform into macrophage-like cells that participate in the inflammatory response, initiate the release of reactive oxygen species (ROS) and cytokines, and ultimately lead to neuron death. Gp91phox (NOX2), a derivative of microglia, can cause neuronal apoptosis through inflammation and the release of ROS. The deficiency of NOX2 can reduce oxidative stress and inflammatory damage [100]. By phosphorylating forkhead box O3 (FoxO3a), maintaining hypochondria membrane permeability, and preventing the release of cytochrome C, Wnt1 limits its transport to microglia to prevent apoptosis and necrosis [101]. Another research has shown that, within a few hours after hypoxia, the expression of inflammatory markers such as tumor necrosis factor (TNF) and IL increases in rats [102]. TNF-*α* can increase glutamate neurotoxicity by inhibiting glutamate uptake, thereby inducing neuronal cell dysfunction. Both IL-1 and TNF-*α* receptor antagonists can attenuate the effect above. The use of pentoxifylline can significantly reduce caspase-3 activity and lighten apoptosis caused by hypoxia [103]. In addition, different regions bear different oxidative stress responses. The increased levels of anti-inflammatory cytokine in the hippocampus and decreased overall levels of M1 and M2 in the lateral medullary medulla (RVLM) could be speculated as a compensatory inhibition of early injury [102].

The article "Insight into the Effects of High-Altitude Hypoxic Exposure on Learning and Memory" was published in 2022. Journal: Oxid Med Cell Longev.

Superoxide dismutase (SOD) functions to maintain an optimal redox status and plays a role in scavenging free radicals. The expression of SOD protein decreases with prolonged hypoxic exposure, and its expression decreases. It is an important contributor to structural damage of the hypothalamic endothelium [86, 104, 105]. Malondialdehyde (MDA) is the end product of the peroxidation of macromolecules such as protein. In general, the SOD to MDA ratio is used to show the cell damage extent by oxygen free radicals and their antioxidant capacity. Some researches have revealed that the hypoxic exposure at an altitude of 7,000 m leads to an increase in the SOD/MDA ratio and that the longer the duration of hypoxic exposure, the greater the SOD/MDA ratio, indicating an increased antioxidant response of the body to some extent [106].

Different cells have different resistance to antioxidant stress. In contrast to neurons, nuclear factor E2-related factor 2 (Nrf2) is highly consistently expressed in astrocytes and has a strong antioxidative capacity [107]. Under the glucose and oxygen deprivation (OGD) model, adenosine, which inhibits inflammation by activating the A1 receptor to protect cell apoptosis, is increased inside and outside neurons. However, astrocytes contribute to extracellular adenosine to a lesser extent than neurons [108]. Studies have demonstrated that hydrogen inhalation reduces hippocampal neuroinflammation by decreasing SOD activity and increasing MDA and B-cell lymphoma-2 (Bcl-2)/Bcl-2 associated X protein (Bax) expression levels [109, 110]. In addition, inhalation of hydrogen-induced BDNF and inhibition of nuclear factor kappa beta (NF-*κ*B) expression may also add contribution to the protective effect [109–111]. Unlike N,N-dimethyltryptamine (DMT), which reduces oxidative stress injury and promotes neuron survival [112], EPO inhibits microglial proliferation and enhances neuron's resistance to inflammatory damage [113, 114].

#### 5.2.2. Effect of Hypoxia on Neurotransmitters and Related Receptors

Acetylcholine (Ach) is a cholinergic transmitter with important physiological functions. Research has revealed that zebrafish reduced levels of acetylcholine in the brain under hypoxic conditions [83]. Advanced studies have found that the phosphorylation of tau (P-tau) in the hippocampus tends to increase during hypoxia [115] and that there is an interaction between P-tau and cholinergic receptors [116]. A negative correlation has been found between changes in P-tau and Ach content [117]. The above results suggest that the impairment of L&M by hypoxia may be associated with an increase in P-tau and a decrease in ACh. The action of hexahydro pyridone derivatives on acetylcholine receptors improves cognitive performance [118].

*γ*-Aminobutyric acid (GABA) is an inhibitory transmitter that is widely distributed in the brain and has many physiological functions. It has a negative regulatory effect in the process of L&M. In the hypoxic environment, the release of GABA increases with the synthesis of rate-limiting enzyme known as glutamate decarboxylase increases (GAD) [119]. And the use of GABA derivative salifen induces hypoxia-induced nerve damage [120].

The article "Insight into the Effects of High-Altitude Hypoxic Exposure on Learning and Memory" was published in 2022. Journal: Oxid Med Cell Longev.

Glutamate (Glu) is the most abundant amino acid in the mammalian brain, and it is also the main excitatory neurotransmitter in the brain, involved in the regulation of L&M and the construction of synapses. Hypoxia leads to activation of defined inositol 1,4,5-triphosphate (insP3). Ca^2+^ then flows into the cytoplasm to activate Scr, leading to a release of large amounts of glutamic acids from microglia, which can be mitigated by vitamin C through blocking the activation of insP3 [121]. Methyl-D-aspartate ionotropic glutamate receptors (NMDARs) are ligand-gated glutamate ion channel, composed of NR1 subunits and NR2 subunits, that plays a critical role in excitatory neurotransmission, brain development, synaptic plasticity related to memory formation, and neurodegenerative diseases in the CNS. The role of NMDARs in the neurological disorder has been most actively studied, especially in neurodegenerative pathologies such as Alzheimer's disease and Parkinson's diseases. It has been demonstrated that NR2A and NR2B are the major subunits of NMDARs in the hippocampus and NR2B subunits are closely related to L&M in mediating some aspects of synaptic function. mRNA and protein levels of the NR2B subunits are significantly reduced in AD and other hippocampal degenerations. Moreover, reducing the expression of NMDARs in NR2B may lead to changes in LTP values [122]. Other studies have found that NMDA-interacting proteins such as postsynaptic density protein 95 (PSD95), postsynaptic density protein 93 (PSD93), and synapse-associated protein 102 (SAP-102) are mainly concentrated in the postsynaptic density (PSD). Under hypoxic exposure, synaptic ras-GTPase activating protein (SynGAP), which is mainly expressed in hippocampal excitatory neurons, is activated by CaMKII and stimulates GTPase activity of Ras, thereby inhibiting the ERK pathway. Hypoxic exposure also increases the expression of NR1 protein in the hippocampal CA1 region and decreases the expression of NR2A and NR2B proteins [106]. Under hypoxic stress, glutamate release increases, leading to overactivity of NMDARs and loss of control of Ca^2+^ influx, ultimately causing neuronal injury and cell death [76]. The ERK signal cascade is closely associated with NMDARs, especially the NR2B subunit. Statins lead to ERK phosphorylation and L&M loss by inhibiting negative regulation of CaMKII/SAP102/SynGAP signaling pathway [123] (Figure 2).

The article "Insight into the Effects of High-Altitude Hypoxic Exposure on Learning and Memory" was published in 2022. Journal: Oxid Med Cell Longev.

#### 5.2.3. Effect of Hypoxia on Energy Metabolism of Nerve Cells

The brain requires very high energy consumption, and it operates with a strict regulatory mechanism to maintain normal neuronal activity. Current research suggests that astrocytes play an important role in energy transfer, production, utilization, and storage, and that glycogen is predominantly found in astrocytes [122]. Glycogen is predominantly found in astrocytes, and in the resting state, astrocytes are responsible for 50% of the glucose metabolism in the mouse brain. This percentage of consumption continues to increase when astrocytes are stimulated [124]. Relative to the classical view, the astrocyte-neuron lactate shuttle (ANLS) hypothesis explains this phenomenon. On the one hand, neuronal activity increases extracellular glutamate, which is transported by the Na^+^ -dependent glutamate transporter and taken up by glial cells. The final metabolic pathway of glutamate includes the conversion of glutamic acid to terephthalic acid via the tricarboxylic acid cycle for oxidation in mitochondria or the reconversion to glutamic acid by taking part in the glutamine-glutamine cycle in neurons. On the other hand, an increase in intracellular Na + concentration activates Na + -K + -ATPase, which increases ATP consumption and glycolysis in astrocytes. Large amounts of lactate produced in astrocytes undergo extracellular release, and extracellular lactate serves as an energy substrate for neurons via monocarboxylate transporter 2 (MCT2). Together with the existence of neurovascular and neurometabolic coupling, these confirm that the complementarity and cooperation of neurons and astrocytes play an important role in neuroenergetics [122].

Astrocytes have a strong glycolytic capacity than neurons [125]. Indeed, both glucose and lactate are energy substrates for neurons. Through conversion, glucose can also enter neurons via glucose transporter 3 (GLUT3) and participate in glycolysis and the pentose pathway [126]. NADPH, the product of the pentose pathway, plays an antioxidant role. In summary, the choice of substrate and how it is used in a balanced manner varies with the environment of the neuron [124, 127, 128]. The ANLS hypothesis has also been debated [129, 130]. The coupling of neurons and astrocytes is important for L&M. Learning leads to a moderate increase in extracellular lactate levels of hippocampal neurons, which reduces the amnesia caused by MCT1 and MCT4 blockade. Neither the inhibition in the expression of the monocarboxylate transporter MCT2 nor the administration of lactate and glucose attenuated amnesia, suggesting that long-term memory is largely dependent on the neuronal uptake of lactate [122], and astrocytes are necessary for the consolidation of glycogen metabolism in L&M cell [131].

The article "Insight into the Effects of High-Altitude Hypoxic Exposure on Learning and Memory" was published in 2022. Journal: Oxid Med Cell Longev.

As the main site of oxygen consumption and energy metabolism, mitochondria must be affected by hypoxia. Hypoxia changes the process of mitochondrial fusion and fission, reduces the stability and oxidative phosphorylation of electron transport chain (ETC) complex proteins, and induces ROS production [132, 133]. Previous research has claimed that ROS-induced Ca^2+^ entry into mitochondria leads to PTP/opening, which further increases ROS production, reduces ETC activity, and leads to cell death [133]. Hypoxia leads to changes in energy metabolism in both neurons and astrocytes (Figure 3). Glucose metabolism disorders play a crucial role in neuronal death after hypoxia cerebral ischemia [134]. In the presence of cerebral ischemia and hypoxia, glycolysis becomes the main pathway of energy generation for neurons, and lactate becomes an important source of energy to maintain neural activity. Furthermore, the expression levels of glucose transporter 1 (GLUT1) and GLUT3 are increased under hypoxia to transport a large amount of glucose involved in glycolysis, which is mediated by HIF-1*α* [134]. In addition, HIF also promotes glycolysis and angiogenesis [135, 136]. Under conditions of impaired metabolic activity in hypoxia, the activity in lactate dehydrogenase, pyruvate kinase, and hexokinase activity is increased. On the flip side, citrate synthase and glutamate dehydrogenase activity are decreased [137]. Moreover, there is direct evidence that prenatal hypoxia and other pathological factors early in life are associated with the antioxidant capacity of neonates [138]. Studies based on rodent models have indicated that chronic hypoxia leads to a decrease in glucose-6-phosphate dehydrogenase (G6PD) activity and NADPH and total glutathione levels that cause neuronal cell apoptosis [139]. Compared to neurons, astrocytes are better able to cope with hypoxia, since astrocytes have glycogen reserves and can rapidly upregulate glucose transporter expression to initiate the glycolysis pathway [140]. Astrocytes are also more resistant to ROS since they have higher levels and higher metallothionein levels. Excitatory amino acid transporter 1 (EAAT1) has been recently found to be involved in glutamate uptake by astrocytes, and the increased expression of MCT4 and EAAT1 could better support neuronal survival under hypoxia stimulation [141]. In the later stage of hypoxia, mutual assistance and cooperation with astrocytes are disrupted due to the massive accumulation of lactate and neuronal toxic damage to neurons [142]. Thereby, researchers have turned their focus on compounds that promote hypochondria energy metabolism to reduce hypoxia-induced cell damage, such as salidroside analog and red hairy Potentilla aquatic extract (RCAE) [143, 144].

The article "Insight into the Effects of High-Altitude Hypoxic Exposure on Learning and Memory" was published in 2022. Journal: Oxid Med Cell Longev.

## 6. Discussion

As increased number of people transport to high altitudes for all reasons in recent years, the effects of altitude environmental exposure on L&M cannot be ignored, and finding strategies to relief or even prevent high altitude-induced CNS disorders is thus of worthy. On the one hand, studies have found that pentoxifylline (PTX), hydrogen, and ginkgolide B can improve L&M by relieving the apoptotic damage of hippocampal neurons [103, 109, 145]. Salidroside analogs could improve the body's oxygen utilization and the total oxyradical scavenging capacity (TOSC) to protect brain function without significant side effects. Ketocoline, glucosamine, and formoterol also reduce memory disorders induced by hypoxia to some extent [83, 146]. On the other hand, epinephrine *α*2 receptor agonists could counteract hypoxia-induced brain disorders, such as clonidine, which decreases ERK1/2 expression levels and phosphorylates CREB and NF-*κ*B and increases NR2B expression in the hippocampus by acting on NMDA receptors to phosphorylate ERK1/2 [147]. Melatonin can also significantly alleviate hypoxia-induced L&M disorders, which may be related to neuron development promotion and inflammation relief [148, 149]. Specific molecular mechanisms, such as by modulating the BDNF/phosphoinositide-3-kinase (PI3K)/AKT pathway to promote hippocampal neurogenesis, may be included [150]. In addition, hypoxic habituation is an important intervention to reduce hypoxic injury. HiHiLo training method is designed to boost participants' hypoxic tolerance in a relative lower altitude environment, such as a plain, and adapts trainees to live in a high-altitude hypoxic environment. Indeed, altitude sickness has been shown to improve as the specific tolerance of the plateau increases [151]. In addition, the use of neural stem cell (NSC) transplantation for the treatment of neurodegenerative diseases has become a research hotspot in recent years [152]. NSCs are cells in the nervous system with the potential of self-renewal and multidifferentiation. Several studies have shown that NSC transplantation can improve learning and memory in rats, which may be related to the process of damaged cell clearance, endogenous neurogenesis stimulation, the ultrastructure of neuron improvement, and the secretion of nutritional factor promotion. Besides, oligodendrocyte transplantation around the ventricle can improve neural behavior defects and reduce myelin basic protein (MBP) deficiency. Although NSC transplantation technology has great potential for application, the treatment mechanism and treatment scheme need to be thoroughly explored, and its application against hypoxic injury remains as a great challenge.

The article "Insight into the Effects of High-Altitude Hypoxic Exposure on Learning and Memory" was published in 2022. Journal: Oxid Med Cell Longev.

About 200 mutated genes have been detected at the cellular and molecular level in studies of mouse cognition, while most mutations caused behavioral deficits. However, the correlation between LTP and L&M is barely positive, possibly due to some other unknown learning-related mechanism. It is obligated to figure out other neurophysiological mechanisms that regulate and interact with LTP in information retrieval and consolidation. To summarize, despite intensive research on the molecular mechanisms underlying hypoxia-induced impairment of L&M capacity, the whole picture of all changes at the molecular and epigenetic levels that shape individual neurobehaviors is far from fully understood. The hippocampus, as the integration center of brain L&M, is the most vital point of hypoxia-induced neurological disorders. Further studies could focus on the mechanisms associated with hypoxia-induced disorders to facilitate the identification of new molecules and genes that could lead to the development of innovative therapies to counteract hypoxia-induced learning and memory deficits.

## Figures and Tables

**Figure 1:** Under normal oxygen, the hydroxylation of two specific proline residues in HIF-1*α* promotes its interaction with VHL E3 ligase. Then, HIF-1*α* proteasome destructs because of ubiquitination. In a hypoxia environment, HIF-1*α* translocates into the nucleus and dimerizes with HIF-1*β* and binds with hypoxia response elements (HREs) to play an important role in adaptive responses to hypoxia stress, linked to numerous signal transduction pathways.

**Figure 2:** In a hypoxia environment, the damage of L&M by hypoxia may be related to an increase in P-tau and a decrease in ACh; with the increase of synthesis of GAD, the release of GABA increases and the use of GABA derivative salifen can improve hypoxia-induced nerve damage. The release of glutamic acid increases, leading to excessive activation of NMDARs and loss of control of Ca^2+^ influx and causing neuronal damage and cell death ultimately.

The article "Insight into the Effects of High-Altitude Hypoxic Exposure on Learning and Memory" was published in 2022. Journal: Oxid Med Cell Longev.

**Figure 3:** The astrocyte-neuron lactate shuttle (ANLS) hypothesis of complementarity and cooperation of neurons and astrocytes and hypoxia can lead to changes in the energy metabolism of neurons and astrocytes.

**Table 1:** The plateau hypoxia environment affects various organs and systems.

System	Result	Study
Respiratory system	High-altitude pulmonary edema	Bhagi et al. [24]
Nervous system	High-altitude cerebral edema	Jensen et al. [27]
	Learning and memory deficits	Cramer et al. [25]
Motor system	Skeletal muscle fiber type change	Chaillou et al. [26]
Digestive system	Duodenal inflammation occurs	Wojtal et al. [28]

## Data Availability

All the data needed for the evaluation of the conclusions of this review are provided in the paper.
